The article "A Web-Based Pharmacological Approach to the Mechanism of Action of Rhizoma Phragmitis and Rhizoma Curcumae in the Treatment of Chronic Atrophic Gastritis" was published in 2022. Journal: Contrast Media Mol Imaging.

# A Web-Based Pharmacological Approach to the Mechanism of Action of Rhizoma Phragmitis and Rhizoma Curcumae in the Treatment of Chronic Atrophic Gastritis

**DOI:** 10.1155/2022/3483774

**Published:** 2022-08-10

**Authors:** Yong Zhi, Shanshan Xie, Changming Shao, Binfang Zeng

**Affiliations:** Xinjiang Medical University, Urumqi 830017, Xinjiang, China

## Abstract

**Objective:**

To analyze and test the effect of *Rhizoma phragmitis* and *Rhizoma curcumae* on the network pharmacology of MAPK (mitogen-activated protein kinase) and TNF (tumor necrosis factor) signaling channels and inflammatory factor target gene regulation in successful modeling of chronic atrophic gastritis rats.

**Methods:**

Rats with chronic atrophic gastritis that were modeled successfully were randomly divided into control and study groups and were treated with conventional western medicine or Rhizoma phragmitis and Rhizoma curcumae, respectively. The pharmacological mechanism of action and efficacy were evaluated.

**Results:**

The treatment efficiency was 76.32% and 97.37% in the control and study group, respectively. After treatment, the serum tumor necrosis factor-*α* (TNF-*α*) and serum malondialdehyde (MDA) levels in the study group were lower than those in the control group and the serum epidermal growth factor (EGF) and superoxide dismutase (SOD) levels in the study group were higher than those in the control group (*P* < 0.05); the pain behavioral scores in the study group were lower than those in the control group, and the free acid quantity and total acid quantity in the study group were higher than those in the control group (*P* < 0.05); the serum MTL index in the study group was higher than that in the control group, and the serum gastrin (GAS) and pepsinogen I (PG I) indices in the study group were lower than those in the control group (*P* < 0.05); the number of 24-hour reflux in the study group was less than that in the control group (*P* < 0.05), and the longest reflux time in the study group was lower than that in the control group (*P* < 0.05).

**Conclusion:**

Based on the network pharmacological results, *Rhizoma phragmitis* and *Rhizoma curcumae* will modulate MAPK, TNF signaling circuits, and inflammatory factor target genes in the chronic atrophic gastritis rat model. This treatment protocol is efficient and beneficial to enhance the gastric function of the chronic atrophic gastritis rat model, while it can alleviate the inflammatory response and significantly reduce the number and duration of reflux, which is a safe and reliable treatment modality.

## 1. Introduction

Chronic atrophic gastritis, a difficult disease of the digestive system, is a long-term damage to the gastric mucosa stimulated by multiple factors, which leads to a decrease in the number of intrinsic glands of the gastric mucosa and even glandular atrophy, often accompanied by nausea, abdominal distension, belching, and in some cases, bile reflux, causing heartburn, bitter mouth, and radiating back pain [1]. The WHO defines chronic atrophic gastritis as a precancerous state of gastric cancer, which should be treated clinically with drugs to reduce the deterioration of the disease. There is no clear conclusion on the pathogenesis of chronic atrophic gastritis, which may be related to genetics, poor lifestyle habits, age, and autoimmunity [2]. From the perspective of Chinese medicine, chronic atrophic gastritis belongs to the category of “fullness” and “gastric pain,” which is closely related to deficiency heat and blockage, and stasis-heat interconnection is the main factor of precancerous lesions, so clearing heat and removing stasis is the key to clinical treatment [3]. The key to clinical treatment is to remove heat and stasis [3].

The article "A Web-Based Pharmacological Approach to the Mechanism of Action of Rhizoma Phragmitis and Rhizoma Curcumae in the Treatment of Chronic Atrophic Gastritis" was published in 2022. Journal: Contrast Media Mol Imaging.

This study was conducted to treat the chronic atrophic gastritis rat model with conventional Western medicine or *Rhizoma phragmitis* and *Rhizoma curcumae* based on systemic pharmacology, which have antibacterial and anti-inflammatory effects and are sweet and cold in taste. *Rhizoma curcumae* longa has blood-breaking and antistatic effects and is warm in nature, bitter, and pungent in taste. Now we would like to analyze the mechanism of *Rhizoma phragmitis* and *Rhizoma curcumae* and investigate the interconnection between chronic atrophic gastritis and pharmacological molecules, target genes, and pathways so as to provide a theoretical basis and a rationale for clinical therapeutic treatment of the disorder, which is presented as mentioned below [4].

## 2. Materials and Methods

### 2.1. General Information

80 SD male rats were adaptively reared for one week and then intervened with free access to 1-methyl-3-nitro-1-nitrosoguanidine deionized water, ranitidine feed, 50° hot saline, and 30° ethanol on alternate days on an empty stomach to construct the disease model of chronic atrophic gastritis. Randomly divided 76 rats were finally modeled successfully into control and study groups, with 38 rats in each group.

### 2.2. Methods

#### 2.2.1. Treatment Methods

*(1) The Control Group.* Ranitidine hydrochloride capsules were purchased from Yunpeng Pharmaceutical Group Co., Ltd., China (No. E210303, specification: 0.15 g). Velase tablets were purchased from LVJINZI Pharmaceutical Group Co., Ltd., China (No. H42022350, specification: 0.2 g). Both medicines were gavaged at a body weight of 0.5 ml/100 g, 1 time/day.

*(2) The Study Group.* TCM decoction-free granules of *Rhizoma phragmitis* and *Rhizoma curcumae* were provided by the Chinese Pharmacy of the First Affiliated Hospital of Xinjiang Medical University. 30 g *Rhizoma phragmitis* and 9 g *Rhizoma curcumae* were decocted with water to 60 ml and then given to the rats by gavage at a body weight of 0.5 ml/100 g, 1 time/day.

The article "A Web-Based Pharmacological Approach to the Mechanism of Action of Rhizoma Phragmitis and Rhizoma Curcumae in the Treatment of Chronic Atrophic Gastritis" was published in 2022. Journal: Contrast Media Mol Imaging.

#### 2.2.2. Material Processing Methods

To obtain the target genes and screen the active ingredients of Rhizoma phragmitis and Rhizoma curcumae, the TCMSP (Traditional Chinese Medicine Systems Pharmacology Database and Analysis Platform) database was applied to search for “*Rhizoma phragmitis*” and “*Rhizoma curcumae*,” the screening conditions were set, and “*Rhizoma phragmitis*” and “*Rhizoma curcumae*” were searched. The target genes and active ingredients of “*Rhizoma curcumae*” were screened, and the relevant target protein stations were searched in the UniProt database, which could obtain the standardized gene names and active ingredients of the Rehmannia-curcuma pairs.

The keywords were searched in the GeneCards database, and the standardized gene names were transformed. After that, the CAG-associated target genes and the active ingredient target genes of “*Rhizoma phragmitis*” and “*Rhizoma curcumae*” were imported simultaneously in VENNY2.1 software, and the Venn diagrams were constructed after mapping, which could be obtained for the cross-gene. Next, to construct the analysis of the disease interaction network, the protein-protein interaction network was constructed by entering the common intersection genes into the String database and the other parameters were set by default. The KEGG pathway results were analyzed by the DAVID database. Network analyzer function was applied to analyze the network characteristics, and the results of the KEGG pathway of Rhizoma phragmitis and Rhizoma curcumae drug combination for chronic atrophic gastritis are shown in Tables 1 and 2.

### 2.3. Observation Indexes

#### 2.3.1. Treatment Effect [5]

Under pathological examination, the symptoms of intestinal epithelial hyperplasia basically disappeared or changed from severe to mild, and gastritis changed from severe to mild to moderate, which was considered significantly effective; the symptoms of intestinal epithelial hyperplasia improved and the level of inflammatory factors decreased, which was considered effective; the symptoms of intestinal epithelial hyperplasia and the degree of gastritis did not improve significantly or worsened, which was considered ineffective. The effective rate = the number of (significantly effective + effective) cases/total cases× 100%.

#### 2.3.2. Inflammatory Factor Profiling [6]

After the last administration of rats in each group, fasted for 24 h and watered, all rats were weighed the next day, anesthetized by intraperitoneal injection of chloral hydrate with 10% hydrate (0.3 ml/kg), and 5 ml blood collection was performed from the abdominal aorta and centrifuged at 3000 r/min for 10 min to obtain serum. The tumor necrosis factor-*α* (TNF-*α*), epidermal growth factor (EGF), malondialdehyde (MDA), and superoxide dismutase (SOD) levels were detected by enzyme-linked immunosorbent assay.

The article "A Web-Based Pharmacological Approach to the Mechanism of Action of Rhizoma Phragmitis and Rhizoma Curcumae in the Treatment of Chronic Atrophic Gastritis" was published in 2022. Journal: Contrast Media Mol Imaging.

#### 2.3.3. Pain Behavioral Score [7]

The rats were placed in an open place, and they were observed and recorded for 5 minutes. Total score = total arching time (s) within 5 minutes × arching grade score. The scoring criteria for hunched back are as follows: 0 points, no hunched posture, exploratory behavior, normal hair color; 1 point, slightly hunched back, exploratory behavior, no hair standing up; 2 points, obvious hunched posture, exploratory behavior reducing, slightly ruffled hair, intermitting abdominal contractions; 3, obviously hunched posture, markedly reducing exploratory behavior, moderately raised hair, intermitting abdominal contractions; and 4, obviously hunched posture, little or no exploratory behavior, the head does not move, on the whole body hair stands up, and the abdomen contracts intermittently. Scores range from 0 points (300 s × 0 points = 0, normal without arching) to 1200 points (300 s ×4 points = 1200, in 300 seconds, continuous arching).

#### 2.3.4. Free Acid Content and Total Acid Content [8]

1 mL of gastric juice supernatant was taken, 1% phenolphthalein indicator was added, it was slowly titrated with 0.01 mol/L NaOH until the pH detector reaches 7.0, the NaOH consumption was recorded as V1, and a 10-fold V1 is the content of free acid contained in the gastric juice; NaOH was continuously added dropwise until the pH detector reaches 8.5, and the NaOH consumption was recorded as V2; V2 is the total acid amount in the gastric juice.

#### 2.3.5. Gastric Function Indicators [9]

Serum gastrin (MTL) level was measured by bis-antibody sandwich method, and serum pepsinogen I (PG I) and gastrin (GAS) levels were measured by enzyme-linked immunosorbent assay.

### 2.4. Statistical Methods

Data were analyzed by the Statistical SPSS22.0 software, if the data conformed to a normal distribution, the measurement data were indicated by means ± standard deviation, and a *T*-test was applied to analyze the data differences between the two groups; the count data were described by the composition ratio and rate, and the chi-square test was applied to analyze the data differences between the two groups. *P* < 0.05 indicated that there were significant variations in the statistical results, and GraphPad Prism8 software was selected to do the graphs in this investigation.

The article "A Web-Based Pharmacological Approach to the Mechanism of Action of Rhizoma Phragmitis and Rhizoma Curcumae in the Treatment of Chronic Atrophic Gastritis" was published in 2022. Journal: Contrast Media Mol Imaging.

## 3. Results

### 3.1. Comparison of Curative Efficiency between the Two Groups

The curative efficiency of the study group was higher than that of the control group (97.37% > 76.32, *P* < 0.05) (see Table 3).

### 3.2. Comparison of the Levels of Inflammatory Factors between the Two Groups

After treatment, TNF-*α* and MDA levels in the study group were lower than those in the control group, and EGF and SOD levels in the study group were higher than those in the control group (*P* < 0.05) (see Table 4 and Figure 1).

### 3.3. Comparison of Pain Behavioral Scores between the Two Groups

Before treatment, there was no noticeable discrepancy in the pain behavioral score between the two groups (*P* > 0.05). After treatment, the pain behavioral scores of the study group were lower than those of the control group (*P* < 0.05) (see Figure 2).

### 3.4. Comparison of Free Acid Quantity and Total Acid Quantity between the Two Groups

Before treatment, there were no significant differences in the free acid quantity and total acid quantity between the two groups (*P* > 0.05), and after treatment, the free acid quantity and total acid quantity of the study group were higher than those of the control group (*P* < 0.05) (see Figure 3).

### 3.5. Comparison of Gastric Function Indexes between the Two Groups

After treatment, the serum MTL index of the study group was higher than that of the control group, and the serum GAS and PG I index of the study group were lower than those of the control group (*P*<0.05) (see Figure 4).

### 3.6. Comparison of the Number of 24 h Reflux and the Longest Reflux Time between the Two Groups

After treatment, compared with the control group, the 24 h reflux number was less and the longest reflux time was shorter in the study group (*P* < 0.05) (see Figure 5).

## 4. Discussion

Chronic atrophic gastritis is a precancerous stage that accelerates the progression from intestinal epithelial metaplasia to gastric cancer. Patients often experience bile reflux and bile-containing duodenal fluid in the stomach, which can seriously damage the gastric mucosa, which in turn can lead to gastric mucosal atrophy [10, 11]. For this reason, effective clinical measures should be developed to reduce the inflammatory response of the gastric mucosa and prevent the deterioration of the disease. In this study, the application of ranitidine hydrochloride capsules and velase tablets western medicine treatment can effectively alleviate the inflammatory response of stomach mucosa in rats with chronic atrophic gastritis, after treatment, rats are prone to drug resistance, while a variety of adverse reactions can occur, and the safety of the treatment is not high [12].

The article "A Web-Based Pharmacological Approach to the Mechanism of Action of Rhizoma Phragmitis and Rhizoma Curcumae in the Treatment of Chronic Atrophic Gastritis" was published in 2022. Journal: Contrast Media Mol Imaging.

There is no clear record of CAG disease name, but according to the symptoms and signs of CAG, TCM attributed it to “epigastric pain, “ruffian,” “gastric ruffian,” and “noisy” belonging to the category of spleen and stomach diseases.

In traditional Chinese medicine, there is no clear record of CAG disease name, but according to the symptoms and signs of CAG, TCM attributed it to “epigastric pain” and “gastric ruffian” belonging to the category of spleen and stomach diseases which can be caused by factors of dietary and emotional disorders [13]. As a result, clinical treatment should be carried out to resolve phlegm, eliminate stasis, regulate qi, and harmonize the stomach [14]. Rhizoma phragmitis and Rhizoma curcumae play important roles in the treatment of chronic atrophic gastritis [15]. In this study, it was concluded by drug similarity (DL), oral bioavailability (OB), and network pharmacological analysis that Rhizoma phragmitis and Rhizoma curcumae contain a total of active ingredients such as quercetin, norberberine, oxidized cork base, palmatine, epiberberine, methylxanthine, and ivy saponin elements, among which the main active ingredients are quercetin, ivy, AR(8), PTGS1(9) RXRA(8), PTGS2(9), SCN5A(8), KCNH2(8), NCOA2(8), and others as the main target protein genes [16]. Rhizoma phragmitis and Rhizoma curcumae can act on the above key target genes, and one active ingredient can correspond to one different target gene, so the acting mechanism of Rhizoma phragmitis and Rhizoma curcumae was very complex [17, 18].

KEGG pathway results showed that Rhizoma phragmitis and Rhizoma curcumae would involve multiple pathways, mainly containing NF-*κ*B signaling pathway, TNF signaling pathway, MAPK signaling pathway, and also serum TNF-*α* and MDA genes [19]. Therefore, Rhizoma phragmitis and Rhizoma curcumae would modulate the genes of corresponding targets of inflammatory factors, which is important for clinical treatment and patient prognosis improvement [20]. A network-based pharmacological analysis revealed that Rhizoma curcumae has the effect of eliminating accumulation of stagnant pain, promoting Qi, and breaking blood and also exerts lipid-regulating, antitumor, antiviral, anti-inflammatory, and analgesic effects. Rhizoma phragmitis is widely used in the clinical treatment of chronic atrophic gastritis and has antipyretic and anti-inflammatory, analgesic, antipyretic, sedative, hypotensive, antioxidant, and hypoglycemic effects [21, 22]. It is said that Rhizoma phragmitis and Rhizoma curcumae have a better anti-inflammatory and analgesic effect by targeting genes on inflammatory factors, and the results of this study are in high agreement with the clinical previous expression results, which provides a promising theoretical basis for the next studies [23, 24]. Gastrointestinal function is impaired in rats with chronic atrophic gastritis, and *Rhizoma phragmitis* and *Rhizoma curcumae* can regulate the body's internal environment, which is conducive to repairing gastric mucosal lesions and enhancing immunity. The results of this study showed that the serum MTL, GAS, and PG I indexes were significantly improved in both groups, and the safety of herbal treatment was higher compared to Western medicine treatment. After treatment, the study group showed significant improvement in all symptoms and shortened reflux time. Therefore, *Rhizoma phragmitis* and *Rhizoma curcumae* can be used clinically as the drugs of choice for chronic atrophic gastritis. However, a more in-depth inquiry is still needed to comprehensively analyze the mechanism of action of *Rhizoma phragmitis* and *Rhizoma curcumae* on chronic atrophic gastritis and refer to more relevant data for subsequent validation.

The article "A Web-Based Pharmacological Approach to the Mechanism of Action of Rhizoma Phragmitis and Rhizoma Curcumae in the Treatment of Chronic Atrophic Gastritis" was published in 2022. Journal: Contrast Media Mol Imaging.

In conclusion, based on the results of network pharmacology, it was shown that *Rhizoma phragmitis* and *Rhizoma curcumae* would regulate MAPK, TNF signaling pathway, and inflammatory factor target genes in rats with chronic atrophic gastritis, and this therapeutic regimen is highly efficient and can improve gastric function, relieve the inflammatory response, and significantly reduce the number and duration of reflux in rats with chronic atrophic gastritis, which is a safe and effective therapeutic modality.

## Figures and Tables

**Figure 1:** Comparison of inflammatory factor levels between the two groups.

**Figure 2:** Comparison of pain behavioral scores between the two groups.

**Figure 3:** Comparison of free acid quantity and total acid quantity between the two groups. *Note.*^#^*P* indicates that the differences in MCS and PCS scores were statistically significant when compared before and after treatment within the group.

**Figure 4:** Comparison of gastric function indexes between the two groups.

**Figure 5:** Comparison of the number of 24 h reflux and the longest reflux time between the two groups.

**Table 1:** Activated ingredients of Rhizoma curcumae drug pairs.

Mol ID	Name of active ingredient	OB (%)	DL
MOL000098	Quercetin	46.42	0.29
MOL002894	Norber berine	35.73	0.72
MOL002904	Oxidized tillerine	36.67	0.83
MOL000785	Palmatine	64.59	0.66
MOL002897	Epiberberine	43.08	0.79
MOL002668	Methylxanthine	45.82	0.88
MOL000296	Ivy saponin element	36.92	0.74

The article "A Web-Based Pharmacological Approach to the Mechanism of Action of Rhizoma Phragmitis and Rhizoma Curcumae in the Treatment of Chronic Atrophic Gastritis" was published in 2022. Journal: Contrast Media Mol Imaging.

**Table 2:** Prediction of disease KEGG pathway by *Rhizoma phragmitis* and *Rhizoma curcumae* drugs.

Signaling pathways	Associated gene number	*P*
NF-*κ*B signaling pathway	12	1.53*E*−09
HIF-1 signaling pathway	12	2.93 *E*−10
Toll-like receptor signaling pathway	13	9.45 *E*−10
FoxO signaling pathway	13	1.48*E*−07
p53 signaling pathway	10	3.05*E*−08
T-cell receptor signaling pathway	12	8.87*E*−08
TNF signaling pathway	20	2.24 E−17
MAPK signaling pathway	16	3.67*E*−07
ErbB signaling pathway	10	3.62*E*−06
NOD-like receptor signaling pathway	11	5.93*E*−09

**Table 3:** The comparison of curative effects between the two groups (n,%).

Group	Number of cases	Invalid	Effective	Significantly effective	Efficient
Control group	38	9 (23.38)	10 (26.31)	19 (50)	76.32%
Study group	38	1 (2.63)	8 (21.05)	29 (76.32)	97.37%
*X* ^2^	—	—	—	—	7.37
*P*	—	—	—	—	<0.01

**Table 4:** Comparison of inflammatory factor levels between the two groups ($\bar{x}\pm s$).

Group	Number of cases	EGF (ng/mL)		TNF-*α* (pg/mL)		SOD (U/mg)		MDA (nmol/mg)	
		Before treatment	After treatment	Before treatment	After treatment	Before treatment	After treatment	Before treatment	After treatment
Control group	38	1.35 ± 0.69	1.52 ± 0.71	30.25 ± 2.08	18.69 ± 1.67	260.35 ± 15.26	358.68 ± 15.49	10.24 ± 2.25	6.12 ± 1.87
Study group	38	1.37 ± 0.72	2.76 ± 0.74	30.21 ± 2.13	14.39 ± 1.21	261.60 ± 16.55	410.27 ± 20.13	10.23 ± 2.32	4.13 ± 1.75
*t*	—	0.139	8.377	0.093	14.446	0.385	14.072	0.021	5.383
*P*	—	0.890	<0.001	0.926	<0.001	0.701	<0.001	0.983	<0.001

## Data Availability

The experimental data used to support the findings of this study are available from the corresponding author upon request.
